# Differences in Outcome and Comparison of Stress and Immune Status in Patients with Recurrent Common Bile Duct Stones after Biliary Tract Surgery Choosing Three Procedures (ERCP, OCBDE, and LCBDE) for Treatment

This article has been retracted.

**DOI:** 10.1155/2022/9197990

**Published:** 2022-01-05

**Authors:** Dong Tan, Yafei Zhang

**Affiliations:** ^1^Department 2 of General Surgery, No. 215 Hospital of Shaanxi Nuclear Industry, Xianyang, Shaanxi, China; ^2^Department of Endoscopy, No. 215 Hospital of Shaanxi Nuclear Industry, Xianyang, Shaanxi, China

## Abstract

**Objective:**

To compare the effect of choosing ERCP, OCBDE, and LCBDE for the treatment of patients with recurrent common bile duct stones after biliary tract surgery.

**Method:**

115 patients with recurrent common bile duct stones after biliary surgery in our hospital were retrospectively analyzed and divided into three groups according to the procedure, 36 patients in the ERCP group, 38 patients in the OCBDE group, and 41 patients in the LCBDE group, and compared the efficacy, stress status, and immune status of the three groups.

**Result:**

The stone removal rates were 91.67%, 97.37%, and 97.56% in the ERCP, OCBDE, and LCBDE groups, respectively (*P* > 0.05). There were statistical differences between the ERCP, OCBDE, and LCBDE groups in terms of operative time, postoperative recovery time of exhaustion, recovery time of defecation, recovery time of feeding, and hospitalization time (*P* < 0.05). The postoperative complication rates were 8.33%, 10.53%, and 7.32% in the ERCP, OCBDE, and LCBDE groups, respectively (*P* > 0.05). The recurrence rates within 1 year after surgery were 2.78%, 7.89%, and 2.44% in the ERCP, OCBDE, and LCBDE groups, respectively (*P* > 0.05).

**Conclusion:**

ERCP has short operative time, short hospital stay, and rapid postoperative recovery. LCBDE has mild trauma, and OCBDE has a wide range of application. Each of the three procedures has its own advantages and shortcomings, and the most appropriate procedure should be selected on the basis of comprehensive evaluation.

## 1. Preface

Biliary lithotripsy is an important method in the clinical treatment of cholelithiasis. Although the surgical results are satisfactory, driven by advances in medical technology, there is still a high risk of recurrent common bile duct stones after surgery, resulting in the need for patients to undergo secondary biliary surgery [1]. Patients with recurrent common bile duct stones after biliary surgery are at a high risk of biliary infection, which is not only acute in onset but also has a high degree of severity, and if not given timely treatment, the patient's life can be directly threatened. The choice of surgical treatment for patients with recurrent choledochal stones after biliary surgery has always been a challenge for clinicians. Since recurrent stones are recurrent stones or residual stones, the location, size, and nature of the stones are different, and the structure of the bile duct and adjacent tissues and organs is also different from that of the first surgery. Therefore, the treatment is significantly more difficult and the surgical risk is greater compared with the first surgery [2, 3]. Currently, the main secondary surgical procedures commonly used for these patients are endoscopic retrograde cholangiopancreatography (ERCP) [4], open common bile duct exploration (OCBDE) [5], and laparoscopic common bile duct exploration (LCBDE) [6], but there is no unified conclusion on which procedure is more effective. In order to provide more guidance on the treatment options for patients with recurrent common bile duct stones after biliary surgery, this study compares the differences in the application of these three procedures in 115 patients, and the results are summarized below.

## 2. Information and Method

### 2.1. Information

We retrospectively analyzed 115 patients with recurrent common bile duct stones after biliary surgery. Inclusion criteria are as follows: patients who were diagnosed with recurrent common bile duct stones by imaging in our hospital, patients who had received at least one previous biliary surgery, patients who had recurrence at least 1 year after the previous surgery, patients who were eligible for secondary surgery, patients who were aware of the study content and signed the consent form, and patients who passed the ethical approval of their hospital. Exclusion criteria are as follows: patients with recurrence at least 1 year after the previous surgery, patients with intrahepatic bile duct stones on preoperative examination, patients with severe underlying diseases that may affect the safety of surgery, patients with contraindications to surgery, and patients who voluntarily requested conservative nonsurgical treatment.

### 2.2. Method

ERCP group: local anesthesia was administered to the pharynx. Diazepam and pethidine were selected for intramuscular injection. The duodenoscope was inserted through the pharynx and entered the duodenum through the esophagus and stomach, and the location of the duodenal papilla was determined with the help of it. The size and shape of the papilla were observed. The catheter was inserted and contrast was injected to determine whether the common bile duct was thickened or not, and the location, number, and size of stones in the common bile duct were observed. The extent of papillotomy was determined according to the size of stones, the results of intraoperative cholangiography, the presence of diverticula, and the relationship between diverticula and papilla. The size of the stones, the intraoperative cholangiogram, the presence of diverticula, and the relationship between diverticula and papillae are used to determine the extent of papillotomy, and balloons and mesh baskets are selected to remove the stones. If the stone is difficult to remove, an internal drain is placed to wait for a second stone extraction. Blood amylase measurement was performed 3 and 6 hours after surgery to observe the symptoms and determine the status of ENBD drainage, and acid suppression and hemostasis were routinely performed.

General anesthesia was given to the OCBDE group. To access the abdomen, an oblique incision was made beneath the right costal border. The liver, common bile duct, and duodenum were revealed after intra-abdominal adhesions were loosened and the neighbouring tissues were entirely liberated. The diameter of the common bile duct was probed and measured, the placement of stones in the bile duct was examined, the presence of stones in the bile duct was verified by puncture, and the bile duct was then incised and probed to ascertain the quantity and size of stones, among other things. To see whether there was any blood congestion, the bottom section of the bile duct was discovered. The T-tube is inserted into the common bile duct if there is no stenosis in the lower half of the duct.

The wound is sutured, and saline is injected to prevent leaking. Roux-en-Y anastomosis of the common bile duct and jejunum was done if the lower section of the common bile duct exhibited stenosis and the stone could not be removed alone. After the procedure, the patient was given gastrointestinal decompression, fasted with food and water, and then, the gastric tube was withdrawn to administer a liquid meal after the gastrointestinal tract function had restored to normal, along with antibiotics to combat infection. LCBDE group: general anesthesia was administered to assist in maintaining a slightly oblique head high and foot low position on the left side. A pneumoperitoneum was established using the four-hole method, intra-abdominal adhesions were loosened after routine abdominal access, and the adjacent tissues were freed to reveal the liver, common bile duct, and duodenum. After confirming the common bile duct by puncture, incisional exploration is performed to evaluate the thickening of the common bile duct and to remove the stone to the maximum extent possible. The intrahepatic bile duct and common bile duct are repeatedly explored with the aid of choledochoscopy. Choledochoscopy can exclude common bile duct stenosis if it is determined that the papilla opening is good, the lithotomy mesh can enter directly into the duodenum, and the intraoperative contrast medium can flow mostly into the duodenum. After determining that there is no stricture in the lower bile duct, the T-tube is placed into the common bile duct and then it is sutured, and saline is injected to make sure there is no leakage. If the lower bile duct showed stenosis, the choledochal jejunojejunostomy was performed as an intermediate open procedure. Postoperatively, the patient was given gastrointestinal decompression, fasted with no food or water, and provided with a liquid diet after the patient's gastrointestinal tract function returned to normal.

### 2.3. Observed Indicator

General information: age, gender, time between previous surgeries, type of previous surgery, and current surgical anesthesia (ASA) classification were counted for the three groups [7].

Stone removal rate: stone removal standard: remove all stones in one operation. Removal rate = number of removal cases/total cases∗100%.

Surgery and postoperative recovery: comparison of the three groups in terms of time to surgery, time to recovery from postoperative exhaustion, time to recovery from defecation, time to return to eating, and time to hospitalization.

Postoperative complications: comparison of postoperative biliary fistula, subcutaneous emphysema, acute cholangitis, papillary hemorrhage, duodenal perforation, common bile duct perforation, and acute cholangitis in the three groups.

Postoperative recurrence: a 1-year follow-up was conducted after the surgery for the three groups, and the recurrence rate of stones during the follow-up period was recorded and compared among the three groups.

### 2.4. Statistical Method

All data were analyzed using SPSS 23.0. [*n*(%)] for count data, *χ*^2^ test, (*x* ± *s*) for measurement data, independent samples *t*-test for between-group comparisons, paired *t*-test for within-group pre-postcomparisons, ANOVA for multipoint comparisons, *F*-test, and GraphPad Prism 8 for graphics; *P* < 0.05 for statistical significance.

## 3. Result

### 3.1. General Information

There was no statistical difference (*P* > 0.05) between the ERCP, OCBDE, and LCBDE groups in terms of the proportion of males to females, mean age, time between previous surgeries, type of previous surgery, and ASA classification of anesthesia for the current surgery (Table 1, Figure 1).

### 3.2. Stone Removal Rate

The stone removal rate in the ERCP group was 91.67 percent, with 33 successful cases and three failed cases out of 36 patients; in the OCBDE group, only 1 stone was not retrieved out of 38 patients, resulting in a stone removal rate of 97.37 percent; and in the LCBDE group, 1 stone was not retrieved out of 41 patients, resulting in a stone removal rate of 97.56 percent. The stone removal rate in the ERCP group was slightly lower than that in the OCBDE and LCBDE groups, but the difference between the three groups was not statistically significant (*P* > 0.05) (Table 2).

### 3.3. Surgery and Postoperative Recovery

The ERCP group had a shorter operative time than the OCBDE and LCBDE groups, with the OCBDE group being shorter than the LCBDE group; the ERCP group had a shorter postoperative hospital stay than the OCBDE and LCBDE groups, with the LCBDE group being shorter than the LCBDE group; and the ERCP group had a shorter postoperative hospital stay than the OCBDE and LCBDE groups.

The ERCP group had a faster postoperative defecation and bowel movement recovery than the OCBDE and LCBDE groups, while the LCBDE group was faster than the OCBDE group. The ERCP group consists of the time to resume eating after surgery was shorter than that in the OCBDE and LCBDE groups, and that in the LCBDE group was shorter than that in the OCBDE group, and the differences were statistically significant (*P* < 0.05) (Figure 2).

### 3.4. Postoperative Complications

In the ERCP group, three patients developed complications after surgery, including one case of subcutaneous emphysema, one case of papillary hemorrhage, and one case of pancreatitis, with a total complication rate of 8.33%; in the OCBDE group, four patients developed complications after surgery, including one case of biliary fistula, one case of acute cholangitis, and two cases of incisional infection, with a total complication rate of 10.53%; in the LCBDE group, three patients had postoperative complications, including one biliary fistula, one acute cholangitis, and one pulmonary infection, with a total complication rate of 7.32%. There was no statistically significant difference in the incidence of postoperative complications among the three groups (*P* > 0.05) (Table 3, Figure 3).

### 3.5. Postoperative Relapse

After surgery, one patient in the ERCP group had recurrence with a recurrence rate of 2.78 percent; one patient in the OCBDE group had recurrence with a recurrence rate of 7.89 percent; and one patient in the LCBDE group had recurrence with a recurrence rate of 2.44 percent. The postoperative recurrence rate did not vary statistically significantly between the three groups (*P* > 0.05) (Table 4, Figure 4).

## 4. Discussion

In comparison to patients treated with surgery on other abdominal organs, a higher percentage of biliary surgery patients need subsequent surgery, which may have a substantial physical and psychological effect on patients and is a significant medical burden [8, 9]. Duodenal diverticulum [10], common bile duct dilatation [11], and surgical injury to the common bile duct [12] are all factors that impact recurrent common bile duct stones following biliary surgery. Age, gender, heredity, metabolism, dietary habits, and obesity, according to other research, may all have a role in the recurrence of common bile duct stones following biliary surgery [2, 13, 14]. Conservative or surgical treatment options are available for individuals with recurrence. Although conservative therapy may reduce surgical damage, it cannot guarantee smooth stone removal, and the recurrence rate following treatment is high [15]. Although invasive, surgical therapy enables for laparoscopy to remove stones and may successfully reduce stone recurrence [16].

Three kinds of operations, ERCP, OCBDE, and LCBDE, were compared in this research, with ERCP achieving quick biliary pressure reduction, efficient infection management, temporary alleviation of illness symptoms, and improved resuscitation efficiency [17]. One patient with acute obstructive purulent cholangitis in the ERCP group was in critical condition and was treated with emergency ERCP+ENBD, which resulted in successful one-time removal of bile duct stones and smooth drainage of purulent bile, which was successfully cured by rehydration and anti-infection treatment after surgery. However, some studies [18] found that ERCP was not an appropriate choice if the patient had excessively hard and large common bile duct stones with a high number of stones or a high degree of stenosis in the lower part of the common bile duct. In this study, there were three cases in the ERCP group in which the stones were not successfully retrieved at one time, one of which was due to the large number of stones and the embedded mesh basket, and the repeated stone retrieval caused papillary edema, which affected the stone retrieval effect; one case was due to the diverticulum papillae, the papillary muscle incision margin was small, and the stones were many and large, which made stone retrieval difficult and ERBD drainage was given for placement; one case was due to the large number of stones and the repeated endoscopic stone retrieval did not retrieve the stones. This study concluded that a comprehensive assessment of the patient is needed before performing ERCP to determine whether there is stenosis in the common bile duct, to determine the location, number, and size of stones, and to remove stones electively after placing drainage if intraoperative fear of difficulty in stone extraction cannot be hard to prevent complications caused by appropriate operation. At the beginning of the clinical application of laparoscopy, patients with a history of biliary surgery had been considered a relative contraindication to LCBDE treatment, and currently, due to the continuous maturation of laparoscopic technology, this contraindication has been eliminated and many successful surgical reports have emerged [19]. For some patients who are too old, obese, unable to tolerate open surgery, or have large stone size, LCBDE treatment can be performed after all preoperative preparatory activities are done [20]. However, one study [21] suggested that an open surgical approach should be chosen if the patient has significant bile duct stenosis and surgical relief is deemed necessary after a clinically aware assessment. In addition, LCBDE should not be chosen if the number of stones is too high resulting in a long extraction time and the patient cannot tolerate a prolonged procedure [22].

The ERCP group had the shortest operative time, which was investigated because this procedure does not require anesthesia or other auxiliary procedures prior to surgery, only a small amount of pain relief and sedative drugs before entering the mirror, making the procedure relatively simple and eliminating the need to wait for anesthesia to wake up after surgery, significantly reducing the operative time. Because this operation does not influence gastrointestinal function, the risk of postoperative complications is low, food may be resumed as soon as feasible, and the therapy is minimally invasive or even noninvasive, allowing for a quicker recovery. The OCBDE group, on the other hand, requires more time for gastrointestinal tract function recovery because the surgical operation has a more obvious impact on gastrointestinal tract function, and the surgery will also cause more obvious damage to the body, and the postoperative incision will take longer to heal, lengthening the hospital stay. There were no significant variations in the frequency of postoperative problems and recurrence rates among the three groups in this research, suggesting that all three treatments offer a high assurance of safety. A study [23] reported the incidence of postoperative pancreatitis in patients with biliary tract stones between 1.8 and 7.2%, and one case of pancreatitis in the ERCP group in this study occurred, which was considered to be due to papilledema obstructing the drainage of pancreatic fluid, or it may be due to excessive amount and speed of contrast injection into the pancreatic duct. A study [24] found that indwelling ENBD drainage significantly reduced the risk of biliary tract infection and postoperative acute pancreatitis. This was confirmed by the medication used in this study.

In summary, ERCP avoids the risk of anesthesia, is highly suitable for elderly patients with chronic diseases and organ failure, does not affect the function of the gastrointestinal tract, has a rapid postoperative recovery, and is highly acceptable to patients, but its long-term efficacy is controversial. LCBDE does not cause significant damage to the biliary tract, and the common bile duct incision is small, which can preserve the integrity of the Oddi sphincter and avoid mechanical damage to the biliary tract caused by laparotomy. The operation has high safety and rapid postoperative recovery, but it has higher requirements on the recipient, and the operation requires a long time, which may be impossible for some patients to tolerate. OCBDE is an open procedure, which is very traumatic and has a long postoperative hospital stay, but it is very suitable for patients with large stones or difficult to remove, those who have undergone multiple surgeries, those who have had damage to the normal structure of the gastrointestinal tract, and those who have to undergo bile-intestinal anastomosis for lower bile duct strictures. The three procedures have their own advantages. All three procedures have their own advantages and shortcomings, and none of them can completely replace the other methods. The present study is inadequate: it was a retrospective study with a large number of subjects, and the results lacked sufficient scientific validity and representativeness; prospective studies with larger sample sizes are needed in the future.

## Figures and Tables

**Figure 1:** Comparison of the interval between previous surgeries. The differences in the interval between previous surgeries after the current stone recurrence in all three groups were not statistically significant (*P* > 0.05).

**Figure 2:** Comparison of surgery and postoperative recovery. Statistical significance (*P* < 0.05) was observed between the three groups for the comparison of (a) surgery time, (b) recovery time from defecation, (c) recovery time from defecation, (d) recovery time from feeding, and (e) hospitalization time. ^∗^*P* < 0.05.

**Figure 3:** Comparison of complication rate among the three groups. Kaplan-Meier curves were plotted for the complication rates between the three groups at the end of surgery, showing no statistically significant differences between the complication rates (*P* > 0.05).

**Figure 4:** Comparison of recurrence rate among the three groups. Kaplan-Meier curves were plotted for the three groups of recurrence rate interval between the end of surgery, showing no statistically significant difference between recurrence rates (*P* > 0.05).

**Table 1:** Comparison of general information between the 3 groups (*x* ± *s*)/[*n*(%)].

Information	ERCP group (*n* = 36)	OCBDE group (*n* = 38)	LCBDE group (*n* = 41)	*t*/*χ*^2^	*P*
Gender					
Male	20 (55.56)	21 (55.26)	23 (56.10)	0.006	0.997
Female	16 (44.44)	17 (44.74)	18 (43.90)		
Age (years)	53.16 ± 18.75	55.68 ± 17.49	53.82 ± 17.24	0.202	0.817
Time between previous surgeries (years)	3.75 ± 1.46	4.06 ± 1.51	3.82 ± 1.49	0.449	0.639
Laparoscopic cholecystectomy	16 (44.44)	18 (47.37)	19 (46.34)		
Open cholecystectomy	7 (19.44)	9 (23.68)	7 (17.07)		
Type of previous surgery					
Bi-II type major gastrectomy	11 (30.56)	10 (26.32)	13 (31.71)	1.090	0.982
Biliary-intestinal anastomosis	2 (5.56)	1 (2.63)	2 (4.88)		
ASA classification					
Grade I	25 (69.44)	23 (60.53)	26 (63.41)	0.665	0.717
Grade II	11 (30.56)	15 (39.47)	15 (36.59)		

**Table 2:** Comparison of stone removal rate after treatment in the three groups (cases, %).

Group	Number of cases	Stone removal	
		Number of clearing cases	Clearance rate
ERCP group	36	33	91.67
OCBDE group	38	37	97.37
LCBDE group	41	40	97.56
*χ* ^2^		1.831	
*P*		0.400	

**Table 3:** Comparison of the occurrence of postoperative complications among the three groups (cases, %).

Types of complications	ERCP group (*n* = 36)	OCBDE group (*n* = 38)	LCBDE group (*n* = 41)	*χ* ^2^/*P*
Biliary fistula	0 (0.00)	1 (2.63)	1 (2.44)	1.521/0.467
Subcutaneous emphysema	1 (2.78)	0 (0.00)	0 (0.00)	2.342/0.310
Acute cholangitis	0 (0.00)	0 (0.00)	1 (2.44)	2.079/0.354
Bleeding nipples	1 (2.78)	0 (0.00)	0 (0.00)	2.342/0.310
Duodenal perforation	0 (0.00)	0 (0.00)	0 (0.00)	/
Perforation of the common bile duct	0 (0.00)	0 (0.00)	0 (0.00)	/
Acute cholangitis	0 (0.00)	1 (2.63)	0 (0.00)	2.233/0.328
Other	1 (2.78)	2 (5.26)	1 (2.44)	0.516/0.773
Total	3 (8.33)	4 (10.53)	3 (7.32)	0.264/0.876

**Table 4:** Comparison of the recurrence rate of stones within 1 year after surgery in the three groups (cases, %).

Grouping	Number of cases	Recurrence	No recurrence
ERCP group	36	1 (2.78)	35 (97.22)
OCBDE group	38	3 (7.89)	35 (92.11)
LCBDE group	41	1 (2.44)	40 (97.56)
*χ* ^2^		1.602	
*P*		0.449	

## Data Availability

The data used to support the findings of this study are included within the article.
